# Research on Multimedia Music Teaching Based on Artificial Intelligence

**DOI:** 10.1155/2022/9730609

**Published:** 2022-08-12

**Authors:** Henghui Ma

**Affiliations:** School of Music and Dance, Ningxia Normal University, Guyuan, China

## Abstract

In order to improve the efficiency of music teaching, this paper constructs a multimedia music teaching system based on artificial intelligence. Moreover, this paper focuses on the technical research of intraframe prediction, intraframe filtering, and transformation technology, respectively proposes the intraframe prediction method based on brightness change and the intraframe filtering technique based on the iterative update, and respectively proposes corresponding optimization algorithms. In addition, this paper proposes intraframe prediction technology based on brightness changes and intraframe filtering technology based on an iterative update, which brings improvements in coding performance, analyzes and verifies the experimental results, and proposes corresponding optimization algorithms, respectively, which saves coding and decoding time. Finally, this paper constructs a corresponding model structure based on actual needs, and analyzes the performance of this model through experimental research. The research results show that the teaching system constructed in this paper has better performance.

## 1. Introduction

At the same time as the progress of science and technology, online education has formed a certain scale, and the music discipline has introduced multimedia technology into music teaching without exception [1]. Since multimedia technology entered music teaching, great changes have taken place in music teaching methods. Some scholars have proposed that the successful use of multimedia teaching makes music teaching more intuitive, interesting, and visual than traditional methods [2]. It can be said that because students can participate interactively, multimedia technology can stimulate students' interest in learning more and make teaching courses alive. In the modern information society, the Internet is not just a simple teaching medium. The Internet can promote education reform [3]. For example, the development of student-centered teaching can fully realize the integration of personalized education, social, school, and family education. Education network application software development, and network design and construction are of great significance to the realization of network education courses. Online education is the main driving force for the establishment of modern information technology based on computer and network technology [4]. Moreover, online education will become the main form of online distance education, an important way to modernize higher education, and will also become a basic lifelong education system. Therefore, it is necessary to make full use of the distance education methods of online education to better achieve the goals of education [5]. In recent years, many schools have established “online education universities,” “distance education,” and modern distance education institutions.

How to introduce modern educational technology and methods into modern distance education to reduce the pressure of shortage of educational resources and existing education shortages, and to adapt to the rapid growth of the demand for technical talents in our country is a new topic [6]. It is necessary to carry out an in-depth and meticulous research and bold exploration of this issue, and to establish a modern distance education system in China that meets the national conditions as soon as possible. The advantage of distance teaching is that it breaks through the limitations of time and space, and increases learning opportunities. It is conducive to expanding the scale of education, reducing teaching costs, sharing excellent teaching resources, realizing curriculum advantages, and building a lifelong education system [7]. Learners can use more abundant teaching and learning resources according to their own time, place, and style, which is also the need of current knowledge and social development [8]. The remote teaching system is used as a remote teaching platform to realize the basic teaching activities of the network live broadcast, so the research of the remote teaching broadcast system becomes very meaningful [9].

## 2. Related Work

For online education, the courseware editing system is a very important part, and it is also an extremely active research direction at home and abroad. Many different experimental and commercial products have appeared one after another. The first category is internationally mature and widely used commercial software such as PowerPoint, Authorware, Dreamweaver, and Flash. Most of this kind of courseware production software adopts the page editing mode, which has a certain degree of independence, and the formed courseware is relatively single and highly targeted, but not flexible enough. At the same time, this type of software has higher requirements for users, requires a certain amount of learning, and is relatively complicated to operate [10].

The second category is a large-scale network teaching system based on the Web. Currently, the most popular systems in the world, with relatively complete functions, are WebCT (Web Course Tools), Blackboard, and Moodle. These three systems can provide teaching staff with various tools and services such as real-time teaching, interactive communication and teaching resource management, support a large number of users, and have a large market share [11]. This article takes WebCT as an example. It is an asynchronous course delivery and management system developed by the Canadian British Columbia Computer Science Department for colleges and universities. It focuses on course content and integrates various related learning tools. Moreover, it can not only publish existing course content on the Internet, but also develop new courses. In recent years, the domestic educational technology community has also begun to pay attention to and independently develop network teaching systems, such as the Chinese version of Blackboard and eyouCT, Longteng multimedia distance education system, Tsinghua network learning platform, Peking University network teaching platform, Nanjing University's sky classroom network teaching system. Although a similar network teaching system has the function of courseware production, its system is huge and the functions are too comprehensive. It tries to cover the entire teaching link of traditional campus education and provide comprehensive support services for online teaching [12]. The third category is an independent network courseware generation system. This type of system or the design of the courseware structure template and wizard mechanism simplifies the steps of network courseware development and greatly reduces the technical threshold of courseware development. Moreover, the courseware-making process is simple, fast, and easy to operate, which is suitable for the development of a large number of network courseware [13, 14].

## 3. The Best Reference Template Selection

### 3.1. Template Definition

As shown in Figure 1, we first use the upper row and left column of the currently encoded image block as the current template and search for a reference template in a certain range of a reconstruction area. Among them, the dark area represents the template. Then, we use the MRSAD (mean-removed sumo absolute differences) of the current template and the searched reference template as a measurement standard to characterize the consistency and matching degree of the current coding block.

(1) $$\begin{array}{c} T_{\text{avg}}=\frac{1}{L}\cdot \sum_{n=0}^{L-1}\left(T_{\text{Pred}}\left(n\right)-T_{\text{Rec}}\left(n\right)\right), \end{array}$$

(2) $$\begin{array}{c} \text{MRSAD}\left(T_{\text{Pred}},T_{\text{Rec}}\right)=\sum_{n=0}^{L-1}\left|T_{\text{Pred}}\left(n\right)-T_{\text{Rec}}\left(n\right)-T_{\text{avg}}\left(n\right)\right|. \end{array}$$

In formula (1), *T*_Rec_ represents the template of the current block to be coded, *T*_Pred_ represents the reference template of the reconstructed block, *T*_avg_ represents the difference between the mean values of *T*_Pred_ and *T*_Rec_, and *L* represents the length of the template. In formula (2), MRSAD(*T*_Pred_, *T*_Rec_) represents the matching degree between *T*_Pred_ and *T*_Rec_.

### 3.2. Template Search

As shown in Figure 1, by searching the reconstructed part of the current frame, the best matching result obtained by matching all the reconstructed reference templates *T*_Rec_ with the current template *T*_Pred_ is the smallest MRSAD between *T*_Rec_ and *T*_Pred_. At this time, *T*_Rec_ is called the optimal reference template *T*_Rec−best_.

(3) $$\begin{array}{c} T_{\text{Rec}-\text{best}}=\text{min}\left\{\text{MRSAD}\left(T_{\text{Pred}},T_{\text{Rec}}\right)\right\},\;T_{\text{Rec}}\in D. \end{array}$$

In the abovementioned formula, *D* represents the search range of the reference template *T*_Rec_ in the reconstructed block of the current frame.

In order to solve the problem of inconsistency between the reference template *T*_Rec_ and the corresponding reconstruction block Rec, we assume that the current template *T*_Pred_ and the reference template *T*_Rec_ approximately satisfy a linear relationship as follows:

(4) $$\begin{array}{c} T_{\text{Pred}}^{\prime }=a\cdot T_{\text{Rec}}+b. \end{array}$$

In the abovementioned formula, *T*_Pred_′ is the approximate representation of the current template *T*_Pred_, a is the scaling factor, and *b* is the compensation factor. In order to get the best fitting effect, we use the least square method, and the problem is transformed into an optimization problem as follows:

(5) $$\begin{array}{c} \text{argmin}\left\|T_{\text{Pred}}-T_{\text{Pred}}^{\prime }\right\|, \end{array}$$

Therefore, the problem is equivalent to

(6) $$\begin{array}{c} \text{argmin}\left\|T_{\text{Pred}}-a\cdot T_{\text{Rec}}-b\right\|. \end{array}$$

It is to find the scaling factor a and the compensation factor *b* to make the abovementioned formula the smallest. a and *b* obtained by solving the optimization problem are as follows:

(7) $$\begin{array}{c} a=\frac{L\cdot \sum \left(T_{\text{Pred}}\left(n\right)\cdot T_{\text{Rec}}\left(n\right)\right)-\sum T_{\text{Pred}}\left(n\right)\cdot \sum T_{\text{Rec}}\left(n\right)}{L\cdot \sum \left(T_{\text{Rec}}\left(n\right)\cdot T_{\text{Rec}}\left(n\right)\right)-\sum T_{\text{Rec}}\left(n\right)\cdot \sum T_{\text{Rec}}\left(n\right)},\\ n=\frac{\sum T_{\text{Pred}}\left(n\right)-a\cdot \sum T_{\text{Rec}}\left(n\right)}{L}. \end{array}$$

The obtained scaling factor a and compensation factor *b* will be used for intraframe brightness compensation prediction.

#### 3.2.1. Intraframe Brightness Compensation Prediction

After obtaining the optimal reference template *m* and the optimal compensation factors a and *b* of the current template, intraframe compensation prediction based on brightness can be performed, and the prediction value of the block to be coded is as follows:

(8) $$\begin{array}{c} \text{Pred}\left(x,y\right)=a\cdot \text{Rec}\left(x,y\right)+b. \end{array}$$

In the abovementioned formula, *x* and *y* represent the position of the pixel with coordinate (*x*, *y*) in the coding block, Pred represents the predicted value of the current block to be coded, and Rec represents the predicted value of the reconstructed block corresponding to the optimal reference template *T*_Rec−best_.

(9) $$\begin{array}{c} \text{Pred}=\frac{1}{N}\cdot \sum_{i=1}^{N}\text{Pred}\left(i\right). \end{array}$$

In order to obtain a better prediction effect, as shown in the abovementioned formula and Figure 2, we selects N sets of optimal candidate templates *T*_Rec_(1), *T*_Rec_(2),…*T*_Rec_(*N*), and linear brightness compensation is performed on each set of candidate templates *T*_Rec_(*i*) to obtain the prediction block Pred(*i*) of the candidate reference template. Finally, the candidate N groups of prediction blocks are averaged to obtain a new prediction block Pred.

When performing intraframe video encoding, the intraframe mode selection at the encoder is determined based on the rate-distortion function, and the mode with the least rate-distortion cost will be selected. The rate-distortion cost function is as follows:

(10) $$\begin{array}{c} \text{min}D\left(R\right),R\leq R_{c}\Leftrightarrow J\left(D,R\right)=D+\lambda \times R. \end{array}$$

That is, the coding distortion is minimized as much as possible at a predetermined code rate. Among them, *R*_*c*_ represents the specified code rate, *R* represents the actual number of bits used to encode the mode, and *D* represents the distortion generated in the mode. In HEVC and H.266, both SSD and SATD are used to express distortion D. The reason is that in intraframe coding, two stages are used to complete the intraframe mode decision process. The first stage is the mode primary selection stage, which uses a low-complexity SATD-based cost function to select N intraprediction modes. The second stage is the mode selection stage, which uses a more complex SSD-based rate-distortion cost function to further select the final intraprediction mode.

(11) $$\begin{array}{c} \text{SSD}=\sum_{i,j}{\left|\text{Orig}\left(i,j\right)-\text{Reco}\left(i,j\right)\right|}^{2}. \end{array}$$

As shown in the abovementioned formula, SSD represents the sum of squares between the errors of the original pixels and the reconstructed pixels.

(12) $$\begin{array}{c} J=\text{SSD}+\lambda_{\text{mode}}\cdot R_{\text{all}}. \end{array}$$

The abovementioned formula represents the rate-distortion function corresponding to SSD. Among them, *λ*_mode_ is the quantization parameter setting, and *R*_all_ represents the number of bits required to encode all the coding information of the current mode, including the following: prediction mode number, division information, and residual coefficient.

Figure 3 shows the SSD-based intra-frame rate-distortion cost calculation process. It can be seen that each mode needs to go through the process of prediction, transform and quantization, inverse quantization and inverse transform, and entropy coding to finally find the optimal prediction mode, which greatly increases the complexity of the encoding end. Therefore, in the first mode selection stage, SATD is used instead of SSD to calculate encoding distortion, which greatly reduces the complexity of the encoding end.

(13) $$\begin{array}{c} \text{Res}\left(i,j\right)=\text{Orig}\left(i,j\right)-\text{Pred}\left(i,j\right),\\ T\left(\text{Res}\right)=H*\text{Res}*H,\\ \text{SATD}=\sum_{i,j}\left|T\left(i,j\right)\right|. \end{array}$$

As shown in the abovementioned formula, SATD first transforms the residual block by the Hada code, and then adds the absolute values of the transformed coefficients. It eliminates the process of transform quantization, inverse quantization and inverse transform, and entropy coding.

(14) $$\begin{array}{c} J=\text{SATD}+\lambda_{\text{mode}}\cdot R_{\text{mode}}. \end{array}$$

The abovementioned formula represents the rate-distortion function corresponding to SATD. *R*_mode_ only calculates the number of bits consumed to encode the current mode.

#### 3.2.2. Intraframe Iterative Filtering Technology

In order to solve the problem of inaccurate prediction of the pixels to be coded in the intraframe prediction far away from the reference pixel, we first analyze the theoretical coding performance of intraframe coding based on the first-order Markov model, compare the theoretical coding performance with the performance of the existing encoder, give a theoretical explanation for the inaccurate prediction of the encoder, and find out the reason for the inaccurate prediction of the encoder. Next, we propose a method based on intraframe iterative filtering, which can effectively improve the performance of the encoder. Finally, considering the implementation complexity of intraframe iterative filtering, a related optimization algorithm is proposed, which greatly reduces the complexity of the encoder and decoder while sacrificing little coding performance.

In HEVC, Chen proposed a theory based on the first-order Gauss–Markov model to analyze the ideal coding performance of intraframe prediction. He pointed out that when performing intraprediction, we need to consider the impact of errors, including quantization errors, noise, and edge pixels. In fact, the availability of reference pixels and errors directly affects the accuracy of intraprediction.

When considering a one-dimensional signal sequence *X*=[*x*_0_, *x*_1_,…,*x*_*N*_]^*T*^, if it is assumed that the signal satisfies the first-order Gauss–Markov chain model with zero mean unit variance, its autocorrelation matrix is as follows:

(15) $$\begin{array}{c} E\left[XX^{T}\right]=\left(\begin{array}{ccccc} 1 & \rho & \rho^{2} & \cdots & \rho^{N}\\ \rho & 1 & \rho & \cdots & \rho^{N-1}\\ \rho^{2} & \rho & 1 & \cdots & \rho^{N-2}\\ \vdots & \vdots & \vdots & \ddots & \vdots \\ \rho^{N} & \rho^{N-1} & \rho^{N-2} & \cdots & 1 \end{array}\right), \end{array}$$

where *ρ* represents the correlation coefficient, which is close to 1. We assume that the first signal sample *x*_0_ in *X* is the reference pixel, which is used to predict *x*_*i*_, *i*=1, ⋯, *N*. As shown in the following formula, there is a weight matrix P which generates a one-dimensional prediction signal $\hat{x}$ as follows:

(16) $$\begin{array}{c} P=\left(\begin{array}{ccccc} 1 & 0 & 0 & \cdots & 0\\ p_{1} & 0 & 0 & \cdots & 0\\ p_{2} & 0 & 0 & \cdots & 0\\ \vdots & \vdots & \vdots & \ddots & \vdots \\ p_{N} & 0 & 0 & \cdots & 0 \end{array}\right), \end{array}$$

where *p*_*i*_, *i*=1,…, *N* represents the weight corresponding to other signals *x*_*i*_, *i*=1,…, *N* predicted by *x*_0_. It can be seen from the abovementioned formula that only the first column of the weight matrix P is nonzero. This is because the predicted values of other signals *x*_*i*_ are only predicted by *x*_0_, as shown in the following formula:

(17) $$\begin{array}{c} {\hat{x}}_{i}=p_{i}x_{0},\\ i=1,\ldots ,N. \end{array}$$

As shown in the following formula, in order to minimize the prediction residual, it is necessary to find the optimal prediction matrix *P*_opt_.

(18) $$\begin{array}{c} P_{\text{opt}}=\text{argminE}\sum_{i=1}^{N}{\left(x_{i}-p_{i}x_{0}\right)}^{2}. \end{array}$$

As shown in the following formula, the optimal weight *p*_*i*_ can be obtained by derivation.

(19) $$\begin{array}{c} P_{i,\text{opt}}=\frac{E\left(x_{i}x_{0}\right)}{E\left(x_{0}x_{0}\right)}. \end{array}$$

Combining the obtained autocorrelation matrix, the optimal prediction weight can be obtained as shown in the following formula.

(20) $$\begin{array}{c} P_{i,\text{opt}}=\rho^{i},\\ i=1,\ldots ,N, \end{array}$$

Therefore, the optimal prediction weight matrix is as follows:

(21) $$\begin{array}{c} P_{\text{opt}}=\left(\begin{array}{ccccc} 1 & 0 & 0 & \cdots & 0\\ \rho^{1} & 0 & 0 & \cdots & 0\\ \rho^{2} & 0 & 0 & \cdots & 0\\ \vdots & \vdots & \vdots & \ddots & \vdots \\ \rho^{N} & 0 & 0 & \cdots & 0 \end{array}\right) \end{array}$$

If we set the residual signal as

(22) $$\begin{array}{c} Y={\left[y_{0},y_{1},\ldots ,y_{N}\right]}^{T}, \end{array}$$

then, the residual matrix is as follows:

(23) $$\begin{array}{c} Y=X-\hat{X}=X-PX=\left(I-P\right)X. \end{array}$$

From this, the autocorrelation matrix of Y can be shown as the following formula:

(24) $$\begin{array}{c} E\left[y_{i}y_{j}\right]=\rho^{\left|i-j\right|}-\rho^{i+j}.\\ i,j=1,\ldots ,N. \end{array}$$

In the one-dimensional signal source distortion-free model, since the reference pixel does not change, the variance of the reference pixel is not considered when calculating the coding performance. The intraframe coding performance can be described as the following formula:

(25) $$\begin{array}{c} G=101{\text{log}}_{10}\left(\frac{{\left(\prod_{i=1}^{N}\sigma_{x_{i}}^{2}\right)}^{1/N}}{{\left(\prod_{i=1}^{N}\sigma_{y_{i}}^{2}\right)}^{1/N}}\right). \end{array}$$

Since the signal has zero mean, the autocorrelation coefficient shown in the following formula is the variance:

(26) $$\begin{array}{c} \sigma_{x_{i}}^{2}=E\left(x_{i}x_{i}\right),\\ \sigma_{y_{i}}^{2}=E\left(y_{i}y_{i}\right). \end{array}$$

It is synthesized to obtain the final optimal coding performance as shown in the following formula:

(27) $$\begin{array}{c} G_{1\;D,opt}=-\frac{10}{N}\sum_{i=1}^{N}{\text{log}}_{10}\left(1-\rho^{2i}\right). \end{array}$$

Similarly, the coding performance of traditional intraprediction can be obtained by formulas. It can be seen from Figure 4 that the black line is the optimal coding performance, and the red line is the coding performance of the traditional prediction method. Here, *ρ*=0.95 and N vary from 4 to 32. It can be seen that the optimal coding performance is far better than that of traditional prediction, and as N increases, the advantage becomes more obvious. The reason is that when N is small, the reference sample point can be very close to other signal samples. When they are very close, the correlation is high. As N increases, it can be found that the approximation effect of the reference sample is worse. The reason is that as the distance increases, the correlation between them becomes smaller. When N is very large, the prediction effect based on traditional prediction methods is poor, and smaller weights should be used to predict the current signal.

## 4. Construction of the Multimedia Music Teaching Model

In order to achieve the purpose of online music teaching, the system intends to use computer technology, communication technology, streaming media technology, and online video live broadcast technology to provide users with a set of online music teaching systems that can be cross-regional, highly shared, and has practical teaching significance. Through field surveys and visits to many places and users, it is determined that the main business characteristics of the system that need to be met are as follows: practical functionality, support for streaming online music appreciation, support for online video live broadcast, provide online teaching and examination functions, and support users consumption management. In addition, it needs to support students to be able to listen to lectures online in real time, independently and flexibly choose past courses, exchange discussions, and online tests. For online teaching, the application of streaming media is also crucial. It needs to compress and transcode music files to achieve the effect of a fast side-by-side and real-time playback. Finally, the system needs to provide powerful system management functions. The online music teaching activities are investigated, and users are divided into three categories: managers, students, and teachers.

The music teaching system based on streaming media is designed with a typical media system, implemented with a standardized network protocol, supports multiple applications such as network video playback, and has strong scalability. The system is composed of streaming media server, web server, storage workstation, video acquisition station, and client. The streaming media server edits, stores, and maintains the video information received from the collection station. The application server executes the web applications of the system. The specific design is shown in Figure 5.

The nonlinear editor can perform special effects rendering, adding letters, and adding watermarks to the recorded video clips. After the video is processed, the video and audio information are transmitted to the video server, and then stored in the video server or directly broadcasted live. The live broadcast processing part of the video server can transfer the analog signal that does not need to be processed to the live broadcast line or store it in the disk. The live broadcast part and the publishing server work together to balance the load of network data. The publishing server is designed and installed in the core computer room of the online music teaching system and publishes the live video information to the student client on the Internet. The student can watch the live course in the live broadcast room of the virtual classroom. At the same time, the video publishing server creates an on-demand service and points the publishing path to the recorded video file in the video storage server for students to review and watch. The system architecture is divided according to the multilayer structure, and the system includes the following: user layer, business logic layer, persistence layer, and data layer. The user layer mainly completes accepting user input and returning the execution result to the user. The business logic layer and the persistence layer are between the user layer and the data layer. They are the bridge between the two and save a large amount of user operation logic. In fact, the database and media library are accessed according to the operation logic. The data layer is responsible for data storage and retrieval, and management of media files.

In the online music teaching system, the transmission of music and tutorials is designed based on streaming media technology. The design of streaming media transmission is based on IP technology, which realizes streaming transmission through grouping and digitization. The realization principle is that the video data is compressed through the compression algorithm, the video data is packaged and transmitted to the client according to the relevant IP protocol, and then, these data packets are combined, and after decompression and decoding, they are restored to the original video data. It realizes the purpose of transmitting video online through the streaming media protocol. The basic process of streaming media transmission in this system is shown in Figure 6.

In the music teaching system, the design of streaming transmission is as follows: (1) when the user chooses to play the streaming media course on the client browser, the client browser will establish HTTP or TCP exchange information with the web server, thereby identifying the required video data from the network data. Then, on the client browser, the streaming media player is started to initialize the acquired video data. The initialized information includes program information, encoding type, and server address. (2) The streaming media player and the streaming media server are based on RTSP (real-time streaming control protocol) to exchange video control information. In addition, the real-time flow control protocol can also support common commands such as play, pause, fast forward, rewind, and record. (3) The streaming media server uses the RTP/UDP protocol to send streaming media data to the streaming media player. When the video data arrives at the client, the streaming media player can decompress and decode the data packet, and then play it. In the transmission and playback of streaming media, two different types of communication protocols, RTP/UDP and RTSP/TCP, can be used to send redirect commands from the server to streaming media players at different addresses.

After constructing the abovementioned model, this paper studies the teaching performance of the model. Combined with the current multimedia music teaching needs, this paper evaluates the teaching efficiency and teaching effect of multimedia music teaching. First, the teaching efficiency is evaluated. The teaching efficiency mainly refers to the speed improvement of the streaming media model compared with the traditional teaching method. Through the analysis of 87 sets of teaching data, the results are shown in Figure 7.

It can be seen from the chart that the model constructed in this paper has a significant effect in improving the efficiency of music teaching. On this basis, this paper evaluates the teaching effect of the model and verifies the teaching effect through the scores of 66 experimental subjects. The results are shown in Figure 8.

From Figure 8, we can see that the multimedia teaching system constructed in this paper performs well in music teaching and has certain practical effects.

## 5. Conclusion

The online music teaching system is designed and implemented based on streaming media technology, and its purpose is to solve the problems encountered in the actual application of online music teaching. When encoding in the rate-distortion mode, considering the directivity of the residual in the current mode, a detailed analysis of the residual energy within the frame is made. When performing transformation, a transformation method based on mode dependence is proposed, which eliminates the traversal process of multicore transformation in H.266 and saves coding time. Moreover, considering the complexity of time coding, this paper does not perform iterative filtering for intraprediction in DC and planar modes, and reduces the number of filtering iterations according to the simulation results to optimize the iterative filtering technology. In addition, this paper conducts research and analysis based on the next-generation video coding standard H.266, and proposes intraframe prediction technology based on brightness changes and intraframe filtering technology based on iterative updating, which will improve coding performance. Finally, this paper verifies the performance of this system through experimental research. The research results show that the model constructed in this paper has a certain effect.

## Figures and Tables

**Figure 1:** Example diagram of intraprediction based on brightness changes.

**Figure 2:** The example diagram of candidate averages for intraprediction based on brightness changes.

**Figure 3:** The calculation process of the SSD-based intraframe rate-distortion cost.

**Figure 4:** Comparison of intraframe performance under the one-dimensional source distortion-free model.

**Figure 5:** System topology.

**Figure 6:** Streaming transmission method.

**Figure 7:** Statistical diagram of the teaching efficiency score.

**Figure 8:** Statistical diagram of the teaching effect score.

## Data Availability

The data used to support the findings of this study are available from the corresponding author upon request.
